# Clinical application of contrast enhanced ultrasound to diagnose benign prostatic hyperplasia

This article has been retracted.

**DOI:** 10.1186/1746-1596-9-133

**Published:** 2014-07-01

**Authors:** Jingfang Shi, Xiaohua Yin, Rong Xu, Yingchun Wang, Lin Jin, Weiwei Gao

**Affiliations:** 1 Department of Ultrasound, Jiading Center Hospital, Shanghai 201800, China; 2 Department of Radiology, Jiading Center Hospital, No.1 Chengbei Road, Jiading District, Shanghai 201800, China

**Keywords:** Contrast enhanced ultrasound, Benign prostatic hyperplasia, Contrast agents

## Abstract

**Abstract:**

**Background**

This study aimed to investigate the clinical significance of contrast enhanced ultrasound (CEUS) in diagnosis of benign prostatic hyperplasia (BPH) through comparing CEUS parameters between BPH and normal person.

**Methods**

A retrospective study of sixty BPH patients (aged 73.5 ± 20.5 years old) and thirty normal controls without prostate diseases (aged 75.3 ± 19.7 years old) who had accepted CEUS detection were performed. Time-intensity curves were obtained for all tests in regions of interest. Images were processed using ACQ software and the following parameters were obtained: arrival time (AT), peak intensity (P), time to peak (TP), area under the curve (AUC), mean transit time (MTT) and extinction time (ET). Differences in inner and outer gland of prostate between BPH and the normal tissue were evaluated.

**Results**

There was a clear boundary between the inner and outer gland of BPH prostate. AT, TP, MTT, ET and P in BPH outer gland were significantly higher than the control group. In inner gland, MTT, ET, AUC and P were also significantly higher than the controls. The accurate rate to diagnose BPH using CEUS was 95.6%, and the sensitivity and specificity were 95.0% and 96.7%, respectively.

**Conclusions**

Among these significantly changed parameters, the increases of MTT, ET and AUC in inner gland and AT, TP in outer gland were most likely related to BPH. These parameters provide an objective visual assessment to diagnosis of BPH.

**Virtual Slides:**

The virtual slide(s) for this article can be found here: http://www.diagnosticpathology.diagnomx.eu/vs/4852383312229155

## Background

Benign prostatic hyperplasia (BPH) is one of the most common benign neoplasms in aging males. Nowadays, with the increased population of aging male, the incidence rate of BPH is also raised [1]. According to epidemiology researches, a dramatic rise in BPH is found in males over the age of 40 and the incidence reached to 50% and 80% in the age of 60 and 80, respectively [2]. Prostate is an abundant blood supply organ and divided into inner and outer gland [3]. The inner gland of prostate (including urethra periurethral zone and transitional areas) is the most predilection site of BPH and sensitive to sex hormone; On the contrary, the outer gland (including central zone and peripheral region) has a lower risk and is insensitive [4].

Nowadays, ultrasonic examination is the most common diagnostic method in BPH. In ultrasonic images, the inner and outer gland of prostate in BPH patients can be clearly observed. Besides, the volume of inner gland in BPH patients is increased significantly, while the outer gland is pressurized to be smaller [5]. Contrast enhanced ultrasound (CEUS) is a technology developed rapidly in recent years. CEUS detection is considered to be an effective and accurate method in BPH diagnosis because of the parameters which make the diagnosis to be visual and objective by distinguishing between normal and hyperplastic tissues [6]. In CEUS, contrast agent is used to enhance the contrast of tissues and blood within the body in medical imaging. The contrast agent greatly improves the sensitivity and accuracy of ultrasound to detect the tissue perfusion [7,8]. Therefore, contrast agent significantly increases the diagnostic potential of CEUS and makes it possible to visualize tumor vascularization [7,8]. Besides, CEUS images have a high spatial and temporal resolution. Several researches have certified this technology has a potential in diagnosis of liver, prostate and other visceral organs tumor [9-12]. But there are few studies on comparison of CEUS in normal prostate and BPH.

In this research, a second-generation ultrasound contrast agent of SonoVue was used to detect ultrasound contrast time-intensity curve in inner and outer gland. The differences and correlations between BPH and normal prostate were studied through contrast CEUS parameters.

## Methods

### Research object

Sixty BPH patients treated by CEUS at Central Hospital of Shanghai Jiading District from May 2009 to October 2012 were studied retrospectively. All of them did not have had prostate surgery and associated with urinary frequency, urinary urgency, or dysuria. Among them, 34 cases were associated with urine retention. They were confirmed not prostate cancer sufferers by transrectal needle biopsy in inner and outer gland. Thirty healthy aging male volunteers without prostate diseases were selected as the normal controls. The age, weight, body mass index (BMI), prostate specific antigen (PSA), hypertension, coronary heart diseases, diabetes and other medical history were recorded (Table 1). All people in the research were told the possible complications of the examination, and signed informed consent. This study was approved by the Shanghai Jiading District Central Hospital Ethics Committee.

**Table 1:** Comparison of baseline data between control group and BPH group

	**Control group(n = 30)**	**BPH group(n = 60)**	***p***
Age(year)	75.3 ± 19.7	73.5 ± 20.5	>0.05
Body weight (Kg)	65.7 ± 10.4	68.5 ± 11.3	>0.05
BMI	22.8	23.2	>0.05
PSA(ng/ml)	2.4	12.6	<0.05
Hypertension(%)	25.7	26.5	>0.05
Diabetes (%)	10.5	9.7	>0.05
Coronary heart disease (%)	13.7	15.4	>0.05

### Research methods

SonoVue (Bracco, Italy), as the contrast agent was mixed with 5 ml physiological saline before a bolus injection of 1 ml mixture to the testing people via ulnar vein. Then a rapid bolus of 5 ml SonoVue-saline mixture was injected to the testing people. Video record was started to detect the contrast agent with time synchronization. The continuing observation was recorded until SonoVue completely subsided. The patient was supine, and CEUS detection was conducted in a cross-section through abdomen with ultrasound diagnostic apparatus (PHILIPS IU22) at probe frequency 2.5-5.0 MHz and mechanical index 0.06.

After CEUS, contrast parameters including arrival time (AT), peak intensity (P), time to peak (TP), area under the curve (AUC), mean transit time (MTT) and extinction time (ET) were analyzed by the ACQ software. Three regions of interest (ROI) of each inner and outer gland were isolated by oval-shaped tracings. The intensity distribution of contrast agent pixels in ROI was used for quantitative analysis, and the mean value in these three ROI was calculated. Besides, a contrast time-intensity curve was also processed. To analyze the CEUS data and make a diagnosis, a single blind method was carried out by 2 experienced examiners. A third experienced examiner was invited to evaluate the data when there was any disagreement.

### Data analysis

The data were expressed as mean ± standard deviation (SD). Statistical analyses were performed with SPSS 13.0 (SPSS Inc., Chicago, USA). Significant differences of contrast parameters between two groups were detected with *T* test. *p* < 0.05 was considered as significant. *p* < 0.01 was considered as highly significant.

## Results

### Basic information of patients

The age of the BPH patients and the controls were respectively 73.5 ± 20.5 years old (n = 60) and 75.3 ± 19.7 years old (n = 30) in the present study. There were no significant difference between the controls and BPH patients in terms of age, body weight, BMI, hypertension, diabetes and coronary heart diseases, but a significant difference in PSA between the two groups (Table 1). According to statistics in BPH patients, the international prostate symptom score (IPSS) was 25.5 ± 4.9, the quality of life score (QOL) was 5.1 ± 0.7, the prostate volume (PV) was 50.6 ± 3.9 ml, the residual urine volume (RUV) was 150.8 ± 47.9 ml, and the maximum urinary flow rate (Qmax) was 8.8 ± 3.3 ml/s.

### CEUS results of the control group and BPH group

CEUS diagnosis in normal prostate and BPH prostate were carried out. Figure 1 showed the CEUS images and the contrast time-intensity curves of the normal prostate and BPH prostate, respectively. Table 2 indicated accurate parameters in normal and BPH prostate.

**Figure 1:** Ultrasound Contrast image and contrast time-intensity curve of normal and A, inner gland in normal; B, Outer gland in normal A1, inner gland in BPH prostate; B1, Outer gland in BPH prostate.

**Table 2:** Data and analyze results of BPH and control group

	**BPH group**		**Control group**	
	**Inner gland**	**Outer gland**	**Inner gland**	**Outer gland**
AT(s)	26.55 ± 2.29	30.84 ± 4.32^☆☆^	27.26 ± 2.10	24.81 ± 2.55
P(%)	53.35 ± 7.70^**#^	36.38 ± 7.20^☆^	44.06 ± 2.57^**^	25.74 ± 6.87
TP(s)	65.69 ± 19.58	58.42 ± 8.48^☆☆^	52.78 ± 4.09^**^	37.16 ± 8.09
AUC(%s)	6135.47 ± 1706.70^**##^	2969.80 ± 1369.06	3987.50 ± 219.66^**^	1993.69 ± 933.34
MTT(s)	98.27 ± 9.12^**##^	77.02 ± 8.50^☆^	76.21 ± 3.10^*^	59.53 ± 14.74
ET(s)	194.89 ± 44.97^##^	159.21 ± 36.04^☆^	127.94 ± 14.52	124.04 ± 13.83

*represents *p* < 0.05 when data of inner gland compared to the outer gland in the same group (**means *p* < 0.01); ^#^represents *p* < 0.05 when inner gland of BPH group compared to the inner gland of Control group (^##^means *p* < 0.01); ^☆^represents *p* < 0.05 when outer gland of BPH group compared to the outer gland of Control group (^☆☆^means *p* < 0.01).

In control group, AT in outer gland was a little shorter than that in inner gland, while the enhanced pattern of inner and outer gland was similar, filling from the peripheral region to the central zone; In 86.7% control group, TP in outer gland was significant shorter than that in the inner gland (*p* < 0.01) and P was also significant lower than the inner gland (*p* < 0.01); ET of the outer gland was shorter than the inner gland without significant difference, the disappeared pattern in outer gland was from central zone to peripheral region. In inner gland, SonoVue was disappeared from peripheral region to urethra periurethral zone; AUC in the outer gland in 93.3% control group was significantly smaller than the inner gland (*p* < 0.01) and MTT was shorter (*p* < 0.05).

In BPH group, the result was different. AT in inner gland was shorter than that in outer gland, but the difference was not significant (*p* > 0.05). The enhanced pattern of inner gland was filling from capsule and urethra periurethral zone to peripheral region, while the outer gland was from capsule to the central zone, there was a clear boundary between the inner and outer gland; TP in inner and outer gland was similar(*p* < 0.01), but P of inner gland was significant higher than the outer gland in 85.0% BPH (*p* < 0.01); ET of the inner gland was longer than that of the outer gland without significant difference, and the SonoVue in inner gland was disappeared from the peripheral region to urethra periurethral zone. Besides, the disappeared pattern in outer gland was uniformly; AUC in 91.7% BPH group exhibited inner gland was significantly larger than the outer gland (*p* < 0.01) and MTT was longer (*p* < 0.01).

### Comparison of CEUS parameters in the control group and BPH group

The CEUS parameters between the BPH and control group were compared (Table 2). In inner gland, there was no significant difference in AT and TP, while significant differences were found in P, AUC, MTT and ET. Compared to the control, the P was significant stronger in BPH group (*p* < 0.05). Besides, the AUC, MTT and ET were significantly higher in BPH group (*p* < 0.01). In outer gland, the AT and TP of BPH were highly significantly longer than the control group (*p* < 0.01); the P, MTT and ET increased significantly in BPH group (*p* < 0.05). Although the AUC was also a bit larger in BPH, but the difference was not significant (*p* > 0.05).

### The diagnostic accuracy

According to the comprehensive analysis of the contrast images and parameters, one case was misdiagnosed to be BPH and three atypical lesions were misdiagnosed to be normal. According to statistics, to diagnose BPH with CEUS, the accurate rate was 95.6% (86/90), the sensitivity was 95.0% (57/60) and the specificity was 96.7% (29/30).

## Discussion

CEUS is a new technology developed rapidly in recent years and beneficial for improving the diagnostic accuracy. SonoVue, a second-generation ultrasound contrast agent, which consists of stabilized microbubbles of a sulphur hexafluoride with remarkable properties [13], is used in this study. It can pass the capillary bed and show the microcirculation [14]. Besides, SonoVue can enhance the echo contrast of blood flow in tissues and conveniently detect the lesion and surrounding tissue perfusion changes through the real-time dynamic observation of the CEUS [15,16]. It is often recommended for a dosage of 2.4 ml [17] or more [18]. In this study, we found 1 ml SonoVue mixture was enough to form a clearly contrast image.

BPH usually occurres in the inner gland of prostate and its pathogenesis is complicated. It is found that the expression levels of angiogenic growth factors (such as vascular endothelial growth factor) in the urine of BPH patients are significantly higher than normal levels, which suggests that angiogenesis is closely related to the incidence of BPH [19,20]. As we know, the main blood-supplied artery for the prostate is bladder artery branched from the internal iliac artery. The bladder artery branches into prostate capsule artery and urethral artery at the junction of the bladder and prostate, which supplies blood to the main part of outer and inner prostate gland, separately [21]. According to the study on radical prostatectomy specimens, the microvessel density in tuberal area is significantly increased in BPH, which prompts that the formation and development of BPH nodules needs increased blood supply [22,23]. Besides, researchers also found abundant neovascularizations were regenerated in BPH gland tissue. Microcirculation in the outer gland is relatively decreased due to increased perfusion pressure from inner gland [22]. In this study, the enhanced pattern in BPH prostate begun to increase in the inner gland and followed by the outer gland, while the disappearance situation was reverse. In addition, significant differences in CEUS parameters between the inner and outer gland were consistent with the former researches [24]. And the P, MTT and ET in inner gland were also longer than the outer gland. These results are closely consistent with the feeding arteries in gland, and indicate CEUS can reflect the distribution and blood flow direction of vascular in BPH accurately and clearly.

When compared with the normal prostate through CEUS, the blood supply of both inner and outer gland in BPH prostate was abundant. This result suggests that not only in the inner gland, the outer gland also have different degrees of proliferation in BPH. Therefore, when CEUS is used to diagnosis the BPH, the inner and outer gland and its corresponding tissue should be compared carefully in order to obtain a scientific and real conclusion. On the other hand, the high level of accuracy, sensitivity and specificity rate of CEUS in diagnosis of BPH further proves that CEUS is an effective means in diagnosis of BPH. However, none of the imaging methods can be regarded as reliable enough on its own, careful attention must to be paid to delicate situations. Prostate biopsy of the biomarkers [25] combined with an entropy-based automated approach to ROI segmentation [26] may provide benefit for diagnosis of BPH or prostate cancer. What’s more, the sample size in the present study is not large enough, so a retrospective study based on larger sample size is needed to confirm the findings in this study in future.

## Conclusions

In conclusion, the information of BPH can be reflected clearly by CEUS parameters. The perfusion condition of contrast agent can indicate the hemodynamic information of the organ which is highly correlated with BPH. Moreover, CEUS can be used to diagnose BPH with a high accuracy, sensitivity and specificity.

## Abbreviations

CEUS: Contrast enhanced ultrasound; BPH: Benign prostatic hyperplasia; AT: Arrival time; P: Peak intensity; TP: Time to peak; AUC: Area under the curve; MTT: Mean transit time; ET: Extinction time; BMI: Body mass index; PSA: Prostate specific antigen; ROI: Regions of interest; IPSS: International prostate symptom score; QOL: Quality of life; VP: Prostate volume; RUV: Residual urine volume.

## Competing interests

The authors declare that they have no competing interests.

## Authors’ contributions

Conceive and design the experiments: JS, XY; Acquire and analyze the data: JS, RX, LJ, WG; Draft the manuscript: YW; Approved the manuscript: XY. All authors read and approved the final manuscript.
